# A transferrin-target magnetic/fluorescent dual-mode probe significantly enhances the diagnosis of non-small cell lung cancer

**DOI:** 10.18632/oncotarget.9482

**Published:** 2016-05-19

**Authors:** Jiali Cai, Bingxin Gu, Fengwen Cao, Shiyuan Liu

**Affiliations:** ^1^ Department of Radiology, Changzheng Hospital, Second Military Medical University, Shanghai, China; ^2^ Department of Nuclear Medicine, Fudan University Shanghai Cancer Center, Shanghai, China; ^3^ Center for Biomedical Imaging, Fudan University, Shanghai, China; ^4^ Department of Oncology, Shanghai Medical College, Fudan University, Shanghai, China; ^5^ Shanghai Engineering Research Center of Molecular Imaging Probes, Shanghai, China; ^6^ School of Biomedical Engineering, Med-X Research Institute, Shanghai Jiao Tong University, Shanghai, China

**Keywords:** molecular imaging, transferrin, MRI/NIRF, non-small cell lung cancer, liver metastasis

## Abstract

To enhance the diagnosis of non-small cell lung cancer (NSCLC), we prepared a dual-modal probe Cy5.5-Tf-Gd-DTPA. Gd-DTPA and near-infrared (NIR) dyes were conjugated to holo-Transferrin (Tf) sequentially, the result of ICP-AES and UV showed 25 Gd ions and 1 Cy5.5 could be loaded per protein, respectively. The calculated longitudinal relaxivity R1 of Cy5.5-Tf-DTPA-Gd was 4.21 mM^−1^S^−1^ per Gd while that of Magnevist (Gd-DTPA) was only 4.02 mM^−1^S^−1^. Confocal laser scanning microscopy and immunohistochemical analyses revealed that the Cy5.5-Tf-DTPA-Gd was localized and accumulated in cytoplasmic vesicles; the cell toxicity assay showed no apparent toxicity. MR and NIR imaging of mice with subcutaneous H1299 xenografte tumors following intravenous injection of Cy5.5-Tf-DTPA-Gd revealed a strong positive contrast of the tumors, which caused a longer lasting enhancement of the MRI signal and fluorescence signal. Taken together, these studies indicate that Cy5.5-Tf-DTPA-Gd could be a good agent for MR/NIRF dual mode applications to detect both tumor in situ and its metastasis.

## INTRODUCTION

Despite advancement of the diagnosis approaches and the development of new molecularly-targeted drugs, lung cancer (most commonly the non-small cell lung cancer, NSCLC) is still the leading cause of cancer related deaths in the United States and worldwide [1]. Early and precise diagnosis of benign and malignant lesions is indispensable for improving current poor prognosis of patients with NSCLC.

Molecular imaging techniques permit direct visualization of target sites and characterization of cellular activity by using contrast agents or molecular probes. The molecular probes can specifically bind to the target location to generate detectable and amplified signals, which have been widely used for tumor diagnosis. Each imaging modality alone has its specific merits and limits. The combination of various techniques can obtain complementary information as well as the sensitivity and specificity data of detection sites, which exhibit synergistic advantages over any modality alone. The magnetic resonance imaging (MRI) offers an excellent capability to examine soft tissues and anatomical references with lack of ionizing radiation and high spatial resolution. Multifarious MRI contrasts, such as superparamagnetic iron oxides, ultrasmall superparamagnetic iron oxides, mangafodipir trisodium, hepatobiliary gadolinium chelates, were developed as imaging enhancers [2, 3]. These chemical compounds contain paramagnetic or superparamagnetic metal ions and can affect the MR-signal properties of surrounding tissues, resulting in enhanced tissue contrast and imaging resolution. The gadolinium-diethylenetriaminepentaacetic acid-based (Gd-DTPA-based) MRI contrast, shortening of T1 relaxation time in tissues and increasing the signal intensity, is the most frequently used clinical magnetic positive contrast so far [2, 4, 5]. However, its rapid clearance, the lack of specificity and the risk of triggering nephrogenic fibrosing dermopathy (NFD) greatly limit its applications [6].

The near-infrared fluorescence (NIRF) dyes are particularly attractive for fluorescence imaging of live animals because of their very little undesired absorption and nonspecific auto-fluorescence. At wavelength of 600 nm and above, the attenuation of penetrating through skin and tissue decays drastically with the increasing of wavelength and reaching the minimum value at 750 nm. Thus, the dyes in this range exhibits an optimal organize penetration. At present, the most commonly used fluorescent NIR dyes are sulfonated carbocyanine dyes (Cy-5, Cy-5.5 and Cy-7) and their derivatives. Dual-modality imaging with NIRF and MRI provides anatomical references in an image by synergistically combining the high spatial resolution and long effective imaging window associated with MR and the high sensitivity of NIRF [7, 8].

The human holo-Transferrin (Tf) is a single poly-peptide glycoprotein consisting of about 679 amino acids, which has an important role in iron transfer in the human body [9]. The transferrin receptor (TfR, also known as CD71) is a transmembrane glycoprotein, consisting of two identical monomers joined by disulfide bonds, with function of mediating the uptake of the iron-chelating protein transferrin [10, 11]. Cancer cells require more iron for their rapid growth and proliferation which results in up-regulation of transferrin receptors in several malignant tumors including lung, brain, breast and colorectal cancers [12]. Transferrin is selected as targeting ligand and as a platform on account of its own natural carboxyl terminal and amino terminal and its characteristics of biodegradable, non-toxic and non-immunogenic. Thus the transferrin, when conjugated with a variety of functional moieties, can be utilized for variety of biomedical applications, such as targeting molecular imaging and drug delivery systems.

In this paper, we describe that the transferrin, when conjugated with paramagnetic metal Gd ions and near-infrared fluorescence dyes Cy5.5, acts as a carrier and vector simultaneously, possessing multi-functionalities and high resolution, and can be utilized for early detection of tumors.

## RESULTS

### Preparation and characterization of the Cy5.5-Tf-DTPA-Gd probe

The procedure for synthesis of the Cy5.5-Tf-DTPA-Gd probe was described in Methods and Materials and schematically presented in Scheme 1. To determine the coupling ratios of transferrin, Cy5.5, and Gd, the concentration of transferrin, the content of Gd, UV–Vis absorption and fluorescence emission spectra were determined by bicinchoninic acid (BCA) method, the inductively coupled plasma optical emission spectrometry (ICP-AES), spectra were obtained on the UV-2550 spectrophotometer and the F-2700 fluorescence spectrophotometer, respectively.

**Scheme 1:** Schematic presentation of the procedure for fabrication of Cy5.5-Tf-DTPA-Gd probe

Three absorption peaks (280 nm, 640 nm and 688 nm) derived from the conjugated Cy5.5-NHS appeared in the UV–vis absorption spectrum of Cy5.5-Tf-DTPA-Gd (Figure 1A-black line). On the other hand, under excitation at 676 nm, the fluorescence emission spectrum of Cy5.5-Tf-DTPA-Gd presented a NIR peak centered at 692 nm (Figure 1A-red line). The absorbance and fluorescence spectra of Cy5.5-Tf-DTPA-Gd were similar to the spectra of free Cy5.5-NHS. The absorption peak at 675 nm (Figure 1B) and the emission peak at 692 nm (Figure 1B) in the ultraviolet–visible (UV–vis) and fluorescence spectra confirmed that Cy5.5 were successfully loaded to transferrin. To quantify the coupling ratio of Cy5.5 per transferrin molecule, the standard curve of absorbance from Cy5.5-NHS was conducted and the data exerted an eminent linear correlation (Figure 1C). With the absorbance of certain concentration of Cy5.5-Tf-DTPA-Gd (obtained from UV), the coupling ratio of Cy5.5 per protein was calculated. Overall, these data indicate that about 25 Gd ions and 1 Cy5.5 molecule were loaded per molecule of transferrin.

**Figure 1:** Characterization of probe **A.** UV-vis adsorption and fluorescence spectra of the probe. Emission curve (red line). Excitation curve (black line). **B.** The absorbance of Cy5.5 (red), Tf (green), Tf-DTPA-Gd (blue) and Cy5.5-Tf-DTPA-Gd (black), confirming the successful immobilization of Cy5.5-NHS on the surface of transferrin. **C.** The absorbance standard curve of Cy5.5-NHS is to quantify the coupling ratio of Cy5.5 per transferrin molecule.

### Magnetic and fluorescence properties of Cy5.5-Tf-DTPA-Gd

The T1 relaxivities of Cy5.5-Tf-DTPA-Gd and Magnevist were increased along with the increasing Gd concentration linearly. The relaxivities of Cy5.5-Tf-DTPA-Gd and Magnevist were 4.21 and 4.02 mM^−1^ s^−1^ respectively (Figure 2A), showing a favorable T1 contrast effect. The fluorescence intensity variation also has a linear relation with the increasing Cy5.5 concentration (Figure 2B). The results indicate that the bio-probe could function as an efficient magnetic/fluorescence imaging contrast.

**Figure 2:** Magnetic and fluorescence properties of Cy5.5-Tf-DTPA-Gd **A.** T1-weighted MR images of Cy5.5-Tf-DTPA-Gd. The T1 relaxivities of Cy5.5-Tf-DTPA-Gd and Magnevist were 4.21 and 4.02 mM^−1^ s^−1^. Upper low: different concentrations of Magnevist (Gd-DTPA). Lower row: different concentrations of Cy5.5-Tf-DTPA-Gd. **B.** The average fluorescence signal intensity of Cy5.5-Tf-DTPA-Gd at different concentrations.

### Cell toxicity studies

Insignificant differences (p > 0.05) in cell viability were observed in the H1229 cells in the absence or presence of the Cy5.5-Tf-DTPA-Gd at a concentration of 100-1000 μg/ml at 37°C for 12 h, 24h and 36h (Figure 3). The decrease in viability after incubation of the cells with the Cy5.5-Tf-DTPA-Gd was less than 5% at the high concentration (700 and 1000 μg/ml), indicating that the probe displays negligible cytotoxicity.

**Figure 3:** In vitro cytotoxicity of Cy5.5-Tf-DTPA-Gd Relative cell viabilities of H1299 cells were measured after being incubated with various doses of Cy5.5-Tf-DTPA-Gd for 12 h, 24 h, and 36 h.

### Specificity and subcellular localization of Cy5.5-Tf-DTPA-Gd

The confocal laser scanning microscopy was employed to examine the intracellular uptake of Cy5.5-Tf-DTPA-Gd in H1229 cells. Red fluorescence dots were observed in the cytoplasm of H1229 cells treated with Cy5.5-Tf-DTPA-Gd, and the signal was increased along with longer incubation time (Figure 4), while the cells pre-incubated with unlabeled transferrin showed no or very weak signal, indicating that Cy5.5-Tf-DTPA-Gd probes were uptaken into the target cells specifically and efficiently.

**Figure 4:** The uptake of Cy5.5-Tf-DTPA-Gd in H1299 cells with different incubation time The incubation transferrin concentration is 100 μg/ml and cultivation time is 5 min (rank 2 and 3) and 30 min (rank 4 and 5). The block groups were pre-incubated with transferrin in a dose of 1 mg/ml for 5 minutes. Cy5.5-Tf-DTPA-Gd (red). DAPI (blue).

### In vivo MR and NIRF imaging

Images obtained from pre-contrast showed no obvious signal contrast difference between tumor and other surrounding organ and tissues. The signal intensity in tumor site started increasing at 5 min after the injection of Cy5.5-Tf-DTPA-Gd and remained steadily high till 24 hour after injection (Figure 5A and 5B). While in the Magnevist treated group, the maximum signal enhancement appeared at 5 min (136.2%) but declined quickly. These observations clearly demonstrate that the tumor signal enhancement by Cy5.5-Tf-DTPA-Gd is obviously higher than that of Magnevist.

**Figure 5:** MR imaging of mice with subcutaneous H1299 cell xenografts **A.** T1-weighted MR images of nude mice at various time points following the i.v. injection of Cy5.5-Tf-DTPA-Gd (upper row), and Magnevist (lower row). The local hyperintensity was visualized using a 7.0 T small-animal MR. White arrows show location of subcutaneous H1299 cell xenografts. **B.** Quantitative analysis of MR images. The average MR relative signal enhancement was measured for each tumor. *p<0.05.

Notably, MR images showed extensive liver metastasis of the xenografted tumors (Figure 6A). Indeed, we found a large sum of macroscopic white tumor metastasis nodules on the surface of liver (Figure 6B). The tumor metastasis nodules were confirmed in (Figure 6A). There was tiny signal contrast between metastasis nodules and normal liver parenchyma in pre-contrast images, the significant difference appeared at 5 min and existed to 24 hour. For mice treated with Magnevist, the inconspicuous contrast was observed at 5 minute point.

**Figure 6:** MR images and HE staining of liver metastasis lung cancer **A.** Obvious liver metastasis (red arrow) in MR images at pre-contrast and different point. (a) Pre-contrast, (b) 5 min, (c) 8 h, (d) 24 h. **B.** Histological images of liver metastasis and H1299 cell xenografted lung cancer. (a) Anatomical picture of liver metastasis (red arrow). (b) The boundary of normal liver tissue and metastasis (c) Representative histological images of normal liver tissue and liver metastasis. (d) H1299 cell xenografted lung cancer.

The fluorescence intensity of targeting group was gradually increasing from 2 hour point and reached peak at 8 hour point and lasted for 24 hour (Figure 7), implying prolonged blood circulation and efficient tumor accumulation of Cy5.5-Tf-DTPA-Gd. Significant fluorescence signal was also observed in liver, spleen, kidney and testis (Figure 8A). In the meantime, the blocking group images show a lower ingestion in tumor as well as other organs. Tumor accumulations of Cy5.5-Tf-DTPA-Gd were 1.35±0.05×10^9^ phto/cm^2^/s in target groups, respectively that of in blocking groups decreased to 0.84±0.06×10^9^ phto/cm^2^/s (p < 0.05) after the competition with free transferrin (Figure 8B). Thus the accumulations could be suppressed after blocked with free transferrin effectively.

**Figure 7:** The near infrared fluorescence imaging in the H1299 cell xenografted lung cancer model Near infrared fluorescence imaging of nude mice following intravenous injection of Cy5.5-Tf-DTPA-Gd (upper row) and blocking with transferrin (lower row) at different time points (0.5, 1, 2, 4, 6, 8, 24 h). The blocking groups were pre-injected with transferrin (10 mg) for 30 minutes in advance. Black arrows show location of subcutaneous H1299 cell xenografts.

**Figure 8:** The bio-distributions of Cy5.5-Tf-DTPA-Gd in subcutanceous xenotransplanted H1299 tumor model **A.** Ex vivo optical imaging of tumor and main organs at 24 h post injection of probe confirmed the in vivo imaging results. **B.** Quantification of the fluorescence intensities in tumors and main organs of the mice injected with Cy5.5-Tf-DTPA-Gd or blocked with transferrin intravenously after accomplishing the near infrared fluorescence imaging. *p<0.05.

The qualitative and quantitative analysis of MRI/NIRF images kept in good concordance, and suggested that tumor accumulation of Cy5.5-Tf-DTPA-Gd was more efficient and the most accumulation culminated at 8 hour post injection.

### Histological analysis

The immunohistochemistry images were closely correlated with the in vivo MRI/NIRF images, and further confirmed that Cy5.5-Tf-DTPA-Gd can accumulate in tumor site with high specificity. The expression level of transferrin receptor in tumor, lung, liver and testis were in accordance with the fluorescence intensities in bio-distribution of Cy5.5-Tf-DTPA-Gd in mice (Figure 9). While further comparison and tissue analysis of the tumor sites and liver confirmed that the focus stem from lung cancer (Figure 6B). The main organs showed no obvious histological and pathological changes with or without the injection of Cy5.5-Tf-DTPA-Gd (Figure 10).

**Figure 9:** NIRF of Cy5.5-Tf-DTPA-Gd probe in tumor tissue and transferrin receptor expression in tumor cells Probe (red), cell nucleus (blue), transferrin receptor (brown). Tumor **A.** lung **B.** liver **C.** testis **D.** Excitation wavelength in fluorescence imaging: DAPI: 340-380 nm; Cy5.5: 650-700 nm.

**Figure 10:** HE staining of main organs with or without injection of Cy5.5-Tf-DTPA-Gd The main organs showed no obvious histological and pathological changes with or without the injection of Cy5.5-Tf-DTPA-Gd. The first and third row (pre-injection), the second and fourth row (post-injection).

## DISCUSSION

In this present study, we developed a tumor-target magnetic/fluorescent dual-modal probe Cy5.5-Tf-DTPA-Gd, which could obtain the comprehensive information of lung cancer sites with the high spatial resolution and excellent sensitivity noninvasively. These data demonstrate that the probe Cy5.5-Tf-DTPA-Gd currently provides the more sensitive detection of tumors in situ and in metastasis sites.

The probe Cy5.5-Tf-DTPA-Gd consists of three portions, transferrin, Gd, and Cy5.5, and each of the components has its own characteristic: 1) transferrin confers the high specificity to its receptor and to avoid the nonspecific effect. Also, the biological compatibility and hypotoxicity makes it a superior agent for biological applications. 2) Gd has an unusually strong hydrogen-proton spin-lattice relaxation effect, which generates the inherent paramagnetic property. After characterized by DTPAa, the heavy-metal toxicity of Gd(III) is decreased on accounting of reducing the space location-obstruct effect and avoiding the direct poison between heavy metal and organism. 3) Cy5.5, in the NIR region, exhibits an increase of tissue penetration and the minimum absorption coefficient of tissue, showing a dominant position in optical imaging of deep tissue and organs. Collectively, these properties make Cy5.5-Tf-DTPA-Gd a good agent formagnetic/fluorescent dual-mode probe.

The quality of contrast enhancement for MR imaging depends on the relaxivity of the contrast agent. The relaxivity R1 observed for Cy5.5-Tf-DTPA-Gd was 4.21 mM^−1^ s^−1^, which is supposed to primarily originate from an increased rotational correlation time associated with the slower rotation of a larger probe in solution [13]. The corresponding T1-weighted images of Cy5.5-Tf-DTPA-Gd demonstrated a continuous increase in brightness as increasing of Gd concentration [14]. This together with the high R1 manifests the applicability of Cy5.5-Tf-DTPA-Gd as an efficient T1 MRI contrast agent. The conjugation of Cy5.5 to transferrin enabled additional fluorescence imaging and generated greater sensitivity in the acquisition of molecular changes in tumor site. The fluorescence emission spectrum of Cy5.5-Tf-DTPA-Gd presented a NIR peak centered at 692 nm (excited at 688 nm). This NIR fluorescence confers Cy5.5-Tf-DTPA-Gd the capability of visualizing tumors in deeper tissues with a low background signal.

When fluorescence materials are used as imaging probes, their intrinsic toxicity limited their use for biological translational research [15–17]. Notably, we did not find any significant cellular toxicity or signs of adverse reaction after probe administration in mice.

In present clinical practice, Gd chelates are still commonly used agents to diagnose neoplastic lesions [18, 19]. These contrast agents are promptly accumulated in vessels of tumor via EPR effect and are retained in extracellular space and subsequently passed into the blood stream, leading to rapid clearance and lack of specificity [2, 20]. The initial accumulation of the Cy5.5-Tf-DTPA-Gd and Gd-DTPA in tumors resulted from the EPR effect rather than specific accumulation [4, 19, 21]. Similar results were obtained with other macromolecular carriers of Gd(III) or Gd-loaded nanoparticles [16]. The active specific accumulation of Cy5.5-Tf-DTPA-Gd occupied the main position by prolonging the blood circulation time, and the distribution of Cy5.5-Tf-DTPA-Gd is mediated by transferrin-Tf receptor interaction. As a consequence, the MR signal intensity and fluorescence intensity in tumor site increases apparently and the maximum values appeared at 8 hour post-administration. High proportions of fluorescence intensity was found in the spleen (0.494±0.037×10^9^phto/cm^2^/s) and liver (2.914±0.023×10^9^phto/cm^2^/s), suggesting that the probe is primarily cleared through the reticuloendothelial system. Interestingly, high intensity is also found in kidney (6.345±0.414×10^9^phto/cm^2^/s), indicating that the probe may also be renal clearable.

Metastasis is a complicated progress with multi-factors and multi-step, coming down to angiogenesis [22], tumor microenvironment [23] and regulated by various cell growth factors [24]. In our study, we established a reliable metastatic model using H1299 lung cancer cells. Extensive metastatic tumor nodules have been consistently found in the liver 15 to 20 days after the initial inoculation. In our study, the significant signal contrast between metastasis nodules and normal liver tissue appeared at 5 min and lasted to 24 hour. The MR images and IHC results verified the existence and origin of the metastasis lesion. In a word, the significant signal contrast between metastasis nodules and normal liver tissue demonstrates that the probe manifests a prominent capacity to identify both primary tumors and metastasis sites.

In summary, we prepared and characterized Cy5.5-Tf-DTPA-Gd, which possessed a high T1 relaxivity and showed a good biocompatibility. In vivo MR and NIRF imaging suggested that Cy5.5-Tf-DTPA-Gd enhanced the tumor contrast and be visually detected due to its accumulation in the tumor site. Given that the transferrin, when conjugated with various functional moieties, can incorporate therapeutic functionalities and further enhance a diverse repertoire of capabilities and it remains to be further studied. Therefore, our Cy5.5-Tf-DTPA-Gd provides a promising platform for developing an MR/NIRF dual-modal biomaterial toward better detection of lung cancer.

## MATERIALS AND METHODS

The human holo-Transferrin (Tf) was purchased from Sigma-Aldrich (St. Louis, Mo, USA). Gd(III) chloride hydrate and DTPAa (diethylenetriaminepentaacetic acid dianhydride) were purchased from J&K Scientific Ltd (Shanghai, China). Cyanine dye 5.5 was purchased from Lumiprobe (Florida, USA). The fetal bovine serum, DMEM (Dulbecco's Modified Eagle Medium) and penicillin and streptomycin were purchased from Gibco (California, USA). CCK-8 (cell-counting kit-8) was purchased from Sigma-Aldrich; DAPI staining resolution (4, 6-diamidino-2-phenylindole) was purchased from Beyotime Inst biotech (Shanghai, China). Human TfR (Transferrin R) Antibody was purchased from R&D system (AF2474, Minnesota, USA).

### Cell lines and animal model

H1299 cells (human non-small lung adenocarcinomic cell line) were obtained from Cell Bank of Chinese Academy of Science (Shanghai, China), and were cultured in DMEM (Gibco, USA) supplemented with 10% fetal bovine serum and 2% penicillin-streptomycin. The cells were incubated at 37°C with 5% CO_2_ in a humid cell incubator.

Five-week-old male Balb/c nude mice were purchased from Lingchang Biotechnology Company Limited, Shanghai, China (Animal Qualification Certification N0. 20130018130073). They were housed in sterile isolated cages with a 12 hour light/dark cycle at constant temperatures of 26°C and had free access to food and water. Animal procedures were carried out according to a protocol approved by the Institutional Animal Care and Use Committee at Second Military Medical University, Shanghai, China. The transferrin receptor overexpressing tumor xenograft model was established by inoculation of 5 × 10^6^ H1299 cells in 100 μL PBS into the subcutaneous tissue of the right hind leg in 5-week old male Balb/c nude mice, which were ready for use when the tumor size reached about 8 mm in diameter.

### Synthesis of Cy5.5-Tf-DTPA-Gd

For synthesis of the probe, 30 mg of holo-transferrin was dissolved in 2 mL of 0.1 M bicarbonate buffer (pH 9.0), then filtered through a 0.2 μm filtration unit. DTPAa (54 mg) was slowly added to the transferrin solution under constant shaking at 550 rpm, and the mixture was incubated at room temperature overnight. A concentration of Cy5.5-NHS was adjusted to 1 mg/mL in DMSO. 400 μL of Cy5.5-NHS solution was added to the mixture above, shaken for 2 h at room temperature. The DTPA and Cy5.5-conjugated transferrin was purified by Amicon Ultra-15 Centrifugal Filter Units (Millipore) through a membrane (cutoff = 10 kDa) and redissolved in 0.1 M citrate buffer (pH = 6.5, 2 mL). Then Cy5.5-Tf-DTPA was reacted with GdCl_3_ (10 mg, 0.038 mmol) in 0.1 M citrate buffer (pH 6.5, 2 mL) for 10 h at room temperature under constant shaking at 550 rpm. The final construct, Cy5.5-Tf-DTPA-Gd was purified by ultrafiltration through a membrane (cutoff = 10 kDa) and redissolved in saline.

### Characterization of the probe

The concentration of transferrin was determined by bicinchoninic acid (BCA) method. The content of Gd was determined on an inductively coupled plasma optical emission spectrometry (ICP-AES, Varian 710-ES, USA). UV–Vis absorption spectra were obtained on a UV-2550 spectrophotometer (Shimadzu, Japan). Fluorescence emission spectra were acquired on an F-2700 fluorescence spectrophotometer (Hitachi, Japan).

The T1 relaxation times of probes at different Gd concentrations were measured with a micro-MRI 7.0 T scanner (Bruker Biospec). The corresponding R1 was calculated from the slope of the linear curve of inverse relaxation time (1/T1) as a function of the Gd concentration. The Cy5.5-Tf-Gd-DTPA was diluted in distilled water at Gd concentration range of 0.075 to 1.2 mM. The samples were transferred to a 96-well plate, and T1 relaxation time was measured. The measurement conditions were T1-weighted echo sequences with the following parameters: echo time (TE) = 8.0ms, T1 number of T1 experiments with repetition time (TR) = 50, 100, 250, 500, 1000, 1500 ms, field of view (FOV) = 58 × 58 mm, matrix = 192×192, slice thickness = 1.0 mm. Images reconstruction and analysis were performed using ParaVision 6.0 (Bruker, Germany).

The fluorescence properties were determined with IVIS® Spectrum Imaging System (PerkinElmer, USA), with the following parameters: excitation peak = 676nm, emission spectra peak = 705 nm. The probe was transferred to a 96 well plate at a transferrin concentration of 50, 100, 150, 200, 250 μg/ml. The fluorescence signal intensity was obtained from the fluorescence image sections of a microplate and the expressed as a mean intensity of selected area.

### Cytotoxicity assay

H1299 cells were seeded in 96-well plates at o density of 5×10^3^ cells per well and cultured for 24 hours. Next, the culture medium was replaced by medium containing Cy5.5-Tf-DTPA-Gd with different transferrin concentrations (0, 100, 300, 500, 700, 1000 μg/ml). After 12, 24 and 36 h of incubating the cells with the probes, the mixture solution 10 μl CCK-8 with 90 μl fresh medium was added to each dishes. The absorbance value (OD) was monitored by a microplate reader at a wavelength of 450 nm. The cell viability was expressed as the percentage of absorbance of the cells incubated with the materials to that of the cells maintained in a normal culture medium. The relative cell viability was calculated according to the following formula: Relative cell viability(%) = (OD_experiment_-OD_blank_)/(OD_0_-OD_blank_) × 100%, where OD_experiment_ is the OD value of different concentrations of Cy5.5-Tf-DTPA-Gd, OD_blank_ is the OD value of blank control, and OD_0_ is the OD value of 0 μg/mL of materials.

### Specificity and subcellular localization of Cy5.5-Tf-DTPA-Gd

Specificity and subcellular localization of the Cy5.5-Tf-DTPA-Gd for TfR was examined by a laser scanning confocal microscopy (Leica TCS-SP5, Leica, Wetzlar, Germany). H1299 cells were harvested and seeded onto confocal dishes at a density of 1×10^5^ cells per well, and were allowed to grow for 24 h. Then, dishes were replaced with the mixture solution of culture medium and Cy5.5-Tf-DTPA-Gd at the concentration of 100μg/ml, while the blocking groups were pre-processed with a saturating dose of free transferrin (1mg/ml) for 5 minutes. After incubated for 5 min and 30 min, cells were fixed with 4% formaldehyde solution for 15 min at room temperature followed by washing with PBS, the cells were stained with DAPI staining solution 15 minutes for nuclear staining.

### In vivo MR imaging

To verify Cy5.5-Tf-DTPA-Gd whether could act as a specific targeting MRI contrast agent for lung cancer, we performed MRI with subcutanceous xenotransplanted tumor model of H1299 in Balb/c nude mice. The T1-weighted imaging was performed using a 7.0 T MRI scanner (Biospec System 70/20, Brucker, Ettlingen, Germany) with a 40 mm diameter mouse body volume coil. Scans were completed before and after injection at 5, 30 min, 1, 2, 4, 6, 8 and 24 hour after tail intravenous injection of Cy5.5-Tf-DTPA-Gd (0.05 mmol Gd/kg). Magnevist was used as control with the same dose. During the MR imaging, mice (n = 3) were anesthetized using gas with a mixture of oxygen and isoflurane (RWD Life Science, China). Heart rate was kept 60-120 times per minute and breath rate was 20-40 beats per minute by changing the ratio of isoflurane/oxygen. The following parameters were used: field of view (FOV) = 45×35 mm; base resolution = 0.176 × 0.137 mm, repetition time (TR) = 400 ms, echo time (TE) = 8 ms, slice thickness = 1.0 mm. The MRI T1 signal intensities (SI) within the regions of interest (ROIs) were measured three times before and after injection of the Cy5.5-Tf-DTPA-Gd. The relative enhancement signal intensity (RESI) was calculated according to the following formula: RESI (%) = SI_contrast_/SI_pre_×100%. The SI_contrast_ is the signal intensity of tumor after the injection at different time points, while the SI_pre_ is that of before the injection of materials.

### In vivo near-infrared imaging and bio-distributions

The nude mice bearing the tumor (6 weeks old, n = 3 per each group) were assessed for Cy5.5 emission at a wavelength of 705 nm after tail intravenous injection of Cy5.5-Tf-DTPA-Gd suspension solution (0.8 mg/kg transferrin of body weight), while the blocking group with a dose of free transferrin (10 mg). During the fluorescence imaging, mice (n = 3) were anesthetized using gas with a mixture of oxygen and isoflurane. The images were taken at different time points (0, 30min, 1, 2, 4, 6, 8 and 24 hour) after intravenous injection of Cy5.5-Tf-DTPA-Gd or Cy5.5-Tf-DTPA-Gd plus free transferrin. The images were obtaining form IVIS^@^ Spectrum Imaging System (PerkinElmer, USA) and were processed by Living Image version 4.3.1 (Caliper Life Sciences, USA).

After NIRF imaging, the mice were sacrificed and the bio-distributions of the Cy5.5-Tf-DTPA-Gd were acquired. Mice were sacrificed and major organs (liver, spleen, kidney, heart, lung, muscle, intestines, testis, bladder, stomach, lymph gland, bone, pancreas and brain) as well as tumor were excised and imaged by IVIS^@^ Spectrum to calculate the average fluorescence intensities within tissues.

### Histological analysis

Tumor tissues and main organs were collected and immediately fixed using 10% formalin solution and paraffin embedded tissues. Ten micrometer sections were prepared and were incubated with a primary human TfR antibody (1:200 dilution, R&D system, USA) in PBS overnight at 4°C and a rabbit anti-goat antibody (1:200 dilution, Skyhobio, Shanghai, China) in combination with streptavidin-horseradish peroxidase (HRP) and the DAB detection system. Untreated sections without any antibody were as negative controls.

For the targeting effect of probe, tumor tissues were collected at the most accumulation time point and fixed with 2.5% glutaraldehyde and stored at −80°C. Frozen samples were cryosectioned by microtome at −20°C into slices of 5 μm thicknesses, and then fixed in cold acetone for 5 min at −20°C. Nonspecific bindings were blocked over 30 min with PBS containing 10% goat serum. The sections were stained with 50 μg/ml of DAPI staining solution in 100 μl PBS for 15 min. The sections were washed with PBS and analyzed under a fluorescent microscope (Nikon Eclipse 50i, H550S).

To confirm the side effects of Cy5.5-Tf-DTPA-Gd in vivo, the tumor-bearing mice were sacrificed immediately after the completion of MRI and NIRF scans at 24 hour points. While the tumor-bearing mice in same batch without disposal act as blank control. Routine paraffin sections and Hematoxylin and Eosin (H&E) staining according to standard clinical pathology protocols were performed.

### Statistical analysis

The data were presented as mean ± SD. values less than 0.05 were considered statistically significant. Means were compared using one-way ANOVA and Student t test. P values less than 0.05 were considered statistically significant.
